# *Melastoma malabathricum* Linn attenuates complete freund’s adjuvant-induced chronic inflammation in Wistar rats via inflammation response

This article has been retracted.

**DOI:** 10.1186/s12906-016-1470-9

**Published:** 2016-12-07

**Authors:** Vikas Kumar, Prakash Chandra Bhatt, Mahfoozur Rahman, Dinesh Kumar Patel, Nikunj Sethi, Atul Kumar, Nikhil Kumar Sachan, Gaurav Kaithwas, F. A. Al-abbasi, Firoz Anwar, Amita Verma

**Affiliations:** 1 Nautral Product Drug Discovery Laboratory, Department of Pharmaceutical Sciences, Faculty of Health Sciences, Sam Higginbottom Institute of Agriculture, Technology & Sciences (Deemed University), Allahabad, -211007 Uttar Pradesh India; 2 Centre for Advanced Research in Pharmaceutical Sciences, Microbial and Pharmaceutical Biotechnology Laboratory, Faculty of Pharmacy Jamia Hamdard, New Delhi, 110062 India; 3 University Institute of Pharmacy, Chhatrapati Shahu Ji Maharaj University, Kanpur, Uttar Pradesh 208024 India; 4 Department of Pharmaceutical Sciences, Dibrugarh University, Dibrugarh, Assam 786001 India; 5 Department of Pharmaceutical Sciences, Babasaheb Bhimrao Ambedkar University (Central University), Vidya Vihar, Rai Bareli Road, Lucknow, 226025 India; 6 Department of Biochemistry, Faculty of Science, King Abdulaziz University, Jeddah, Saudi Arabia; 7 Bio-organic & Medicinal Chemistry Research Laboratory, Department of Pharmaceutical Sciences, Faculty of Health Sciences, Sam Higginbottom Institute of Agriculture, technology & Sciences (Deemed University), Allahabad, -211007 Uttar Pradesh India

**Keywords:** *Melastoma malabathricum Linn*, Complete Freund’s Adjuvant, Pro-inflammatory mediator, Inflammatory mediator

## Abstract

**Background:**

Natural products use for arthritis treatment is gaining importance in the medical worldt. Various studies reports medical importance of *Melastoma malabathricum Linn*. (*MM*) (Melastomataceae), also known as “putki,” has a broad range of health benefits, for its free radical scavenging constituents. The current investigation scrutinizes the antioxidant and anti-inflammatory effect of *MM* against adjuvant-induced arthritis in experimental rats.

**Methods:**

High-performance thin layer chromatography (HPTLC) was used for estimation of phytochemical-constituents present in the *MM* extract. Protective effect of *MM* extract in Wistar rats was estimated using CFA-induced model. The rats were divided into different groups with six rats in each group. All animals received oral administration of *MM* and indomethacin for 28 days. The body weight and arthritic score were scrutinized at regular intervals. At the end of experimental protocol, the rats were sacrificed, and blood samples were used for antioxidant, hematological parameters, pro-inflammatory and inflammatory mediator, respectively. Histopathological observation was used to evaluate the protective effect of *MM* extract.

**Result & discussion:**

Current study confirmed the preventive effect of *MM* against adjuvant-induced paw edema, paw redness and arthritic progression. *MM* significantly (*P* < 0.001) modulated the oxidative stress parameters as well as hematological parameter induced by CFA. The result also altered the distorted level of proinflammatory mediators and inflammatory mediator, which further reinforce the implication of *MM* in CFA induced arthritis. Histological analyses of joints of rats showed a reduction in the synovial hyperplasia and mononuclear infiltration in the *MM* treated group which provides evidence for the antiarthritic effect of *MM*.

**Conclusion:**

From above parameters our study states that the *MM* is capable of restraining the alteration produced via adjuvant-induced arthritis in aminals. The repressing effect of *MM* could be attributed, at least in part, to antioxidant, hematological and anti-inflammatory effect.

**Graphical abstract:**

Figure Caption: *Melastoma Malabathricum* Linn Attenuates Complete Freund’s Adjuvant-Induced Chronic Inflammation in Wistar rats by Inflammation Response

## Background

Rheumatoid arthritis (RA) is a chronic immune-mediated inflammatory disease, which finally results in damage of ligaments, peripheral joints and tendons. RA affects around 1% people in developed countries [1–5]. RA is further defined as the inflammatory condition of joints, which produces the pain, immobility and inflamed condition with excess deposition of synovial fluid (accumulation of polymorphonuclear leukocytes) [6, 7].. NSAIDs (Nonsteroidal anti-inflammatory drugs) are well established class of drugs used by many physicians on their patients as a first line antiarthritic drug, but they have side effects such as gastric erosion, ulceration, liver toxicity, inhibition of platelet activation and gastrointestinal hemorrhage, which consequently result in increased risk of hemorrhage [8, 9]. A lot of drugs have been developed for the treatment of RA over the past two decades, but researchers are still in search for more specific drugs with minimum side effects. Researchers were able to explain the one of the herbal formulation piascledine, which is the mixture of avocado and soybean oils sfor relief of inflammatory arthritis symptoms. Several other small anti-inflammatory compounds isolated from natural sources have been scrutinized for the development of new lead molecule in the treatments for RA, but scientific data of their antiarthritic efficacy is still deficient and need more thorough study.

*Melastoma malabathricum Linn.* (Melastomataceae) (*MM*), commonly known as Phutki in India, is a branched shrub available in subcontinent, especially in northeastern region. Traditionally, its leaves are chewed and applied to cuts and wounds for their coagulating properties. The leaves are used to treat hemorrhoid, dysentery, diarrhea and to prevent scarring from the pox. The shoots are used as a toothbrush for toothache,. Leaves and roots powder can be applied to pox scars and wounds to expedite the healing process or to alleviate the uneasiness of hemorrhoids. Flowers are used to treat stomach-ache [10, 11, 12]. *MM* plant has been utilized in the treatment of inflammation and rheumatism by the local people in Dibrugarh district, Assam. The plant is rich source of different chemical constituents such as α-amyrin, patriscabatine and auranamide [13], kaempferol-3-O-(2”,6”-di-O-p-trans-coumaroyl)glucoside, quercitrin, Mefloquine, (+) 3,4-Dehydroproline amide, 2-(3,5-Diphenyl-pyrazol-1-yl) benzothiazole, Kaempferol, Kaempferol-3-O-(2”, 6”-di-O-p-trans-coumaroyl)-β-glucopyranoside [14, 52].

Researchers have proved the antinociceptive, anti-inflammatory, antipyretic [15, 16], antidiarrhoeal [17], antimicrobial [18], antiproliferative and antioxidant [19], antiulcer activity [20], acute toxicity evaluation, antibacterial, antioxidant and immunomodulatory effects and hepatoprotective activity [21, 22] of the plant. However, this plant is not scientifically explored for its antiarthritic activity. Hence, efforts were made by the authors to screen the antiarthritic potential of *MM*.

## Methods

### Drugs and chemicals

CFA was procured from Sigma Chemical Company, USA and Indomethacin from Micro Lab Pvt. Ltd., India. Rest of the chemicals used in the experimental protocol was purchased as an analytical grade from the approved vendor.

### Plant material

*MM* leaves were collected from the Herbal Garden, Dibrugarh University, Dibrugarh, Assam and authenticated by the Botanical Survey of India, Shillong and specimen voucher of plant sample was deposited for future reference.

### Preparation of extracts

*MM* leaves were thoroughly cleaned with tap water to eliminate extemporaneous matter and dried in the shade. The dried *MM* (1 kg) leaves samples were exhaustively extracted with methanol in Soxhlet extractor for 72 h [23, 24]. The extract was filtered using the Whatman filter paper and the filtrate was concentrated under reduced pressure at low temperature. The extract was stored at 4 °C until further use. Before experimentation, *MM* extract was freshly prepared by dissolved in 1% carboxyl methyl cellulose (CMC) for experimental study.

### Chromatography experiment

Pre-coated silica gel plate 60 F254 with a width (6 mm band) used for the HPTLC. Camag microliter syringe with a Linomat 5 applicator was used for injecting the sample over the plate under a flow of Nitrogen gas. The mobile phase {Hexane/ethyl acetate/formic acid (5:4:1, v/v/v)} was used in linear ascending development. The saturation time for mobile phase was about 20 min in saturation chamber to obtain the best results of tested and reference samples at room temperature (27 ± 20 °C) with 50% ± 2 relative humidity. Finally, the TLC (Thin layer chromatography) plate was dried at room temperature and the TLC plate image was developed at the distance of up to 80 mm length.

### HPTLC (High-Performance Thin Layer Chromatography) photo-densitometry

HPTLC study of *MM* extract was carried out according to reported method of Kumar et al. with minor modification [25]. Quercetin (10 mg) was dissolved in 10 mL of methanol for preparing the standard solution and *MM* (2.0 g) extract solution was dissolved in 50 mL of methanol and was subjected to filtration using the Whatman filter paper. The filtrate was completely evaporated under reduced pressure and the obtained remains were re-dissolved in 1 mL of methanol. The prepared solution of quercetin and *MM* extract was carefully spotted on the precoated TLC plates using Camag microliter syringe with constant application 150 nL/s.

### Molecular docking studies

The molecular docking study was performed on cyclooxygenase 2 (3D structure) complex enzyme using Maestro 9.0 program (Schrodinger Inc. USA) by 64 bits operating systems under Windows 7 with an HCl computer [Intel (R) Core (TM) i5-2400 CPU @ 3.10 GHz, 8GB memory]. The molecular docking study was performed on enzymes cyclooxygenase, which was taken from the protein data bank (PDB ID: 1cx2). The protein is having the 96% similarity with the human cell enzyme with all the active site residues. Before performing the molecular docking, the enzyme structure was scrutinized for missing bonds, atoms and contacts. All residues and water molecules were manually removed from the structure. The grid box was used for the estimation of the active site of the protein. The minimum energy was selected and used an energy minimization.

### Animals

Swiss albino adult Wistar rats (weighing 150–220 g; both sexes, kept six per cage) were obtained from the departmental animal house and were used according to departmental ethical committee and care of animals (National Institutes of Health). The animals were housed in the animal house under standard conditions (relative humidity (55 ± 10%), temperature (23 ± 1 °C), 12 h/12 h light/dark cycles) they received the standard pellet diet and water *ad libitum*.

### Acute toxicity study of *MM*

Oral acute toxicity study of *MM* extract was performed according to the reported method of Kumar et al. with minor modifications [25]. Swiss albino Wistar rats of both sexes (weighing 100 to 220 g, body weight) were used for the experimental purpose. The rats were ravenous overnight and divided into the four groups (each group of rats contained three male and three female rats): Group I: (normal control) treated with vehicle only (1 mL water) and Group II (tested) received *MM* (0.5 g/kg); Group III received *MM* (1.0 g/kg, body weight (b.w.)) and Group IV received *MM* (2.0 g/kg b.w.), respectively. All group animals were examined for 24 h, for the confirmation of signs and symptoms of autonomic, neurological and behavioral changes [26].

### Sub acute toxicity study of *MM*

Swiss albino Wistar rats (weighing 100 to 220 g; both male and female) were randomly selected randomly for the study. The animals were divided into four groups and each group contains animals (five male and five female): Group I- normal controls received vehicle (1 mL water); Group II- treated *MM* (500 mg/kg b.w.); Group III- treated *MM* (1000 mg/kg b.w.); Group IV- treated *MM* (2000 mg/kg b.w.). All animals treated with predetermined oral treatment and *MM* extract which was suspended in distilled water.

All group animals were observed for adverse reactions, side effects, mortality and any other changes at end of the sub acute toxicity study. The food consumption, water intake and body weight of all group animals were scrutinized at regular intervals. At the end of protocol nimals were sacrificed by cervical dislocation using the anesthesia condition, all the vital organs of animals were scrutinized visibly for evidence of any morphological deformity and blood samples of all group animals were collected and were used for the estimation of serum biochemistry like RBC (red blood cells), WBC (white blood cells), Hb (hemoglobin) and platelets levels and the biochemical parameters like AST (Aspartate aminotransferase), ALP (Alkaline phosphatase), ALT (Alanine transaminase), total cholesterol, LDL (Low-density lipoprotein), VLDL (Very low-density lipoprotein), HDL (High-density lipoprotein), triglyceride, bilirubin, albumin, creatinine, total protein and serum urea were also estimated [53]. The vital organs such as kidney, heart and liver were excised, removed and weighed. Samples of extraneous tissues were removed, fixed in 10% formalin and dehydrated for histopathological examinations [27].

### Oral administration of drugs

The flexible metal rodent feeding tube was used for oral administration of tested and reference drugs. Mis-feeding of tested and reference drugs into trachea was perceived by signs of an irregular breathing pattern, irritation and choking. When the misfeeding transpired (less than 5% of all feedings), the rats were carefully observed for their revival [28].

### Complete Freund’s Adjuvant-induced arthritis in rats

The rats were divided into six groups (each group 6 rats). Group I was treated with vehicle (1% (*w/v*) CMC); II received CFA; III received CFA + *MM* (100 mg/kg); IV received CFA + *MM* (250 mg/kg); V received CFA + *MM* (500 mg/kg) and Group VI received CFA + indomethacin (10 mg/kg). CFA (0.5% *w/v*) was inducted into the sup-planter region of left hind paws to induced the arthritis. All the animals received the predetermined treatment till 28 days [29, 30] with paw edema of rats subjected to scrutinized at a regular interval using the screw gauge micrometer [31].

### Evaluation of arthritis swelling

The joint swelling (arthritis index) was evaluated by the reported method of Kumar et al. [25] with minor modifications. The arthritic index was assessed on scale 0–4, 0: no change, 1: mild swelling and erythema of limb, 2: erythema of limb and moderate swelling, 3: erythema of limb and coarse swelling, 4: the inability of limb and gross deformity. The score of the four limbs was counted. Score more than one, confirmed arthritis and limited score of arthritis was set to 16. The arthritis score day of onset and frequency of arthritis was also recorded [32].

### Blood and tissue sampling

Rats of all groups were sacrificed on 29^th^ day, and blood samples were collected in test tubes with anticoagulation agent. The collected blood samples were centrifuged at 15,000 rpm, and the serums were obtained for the estimation of biochemical parameters.

### Estimation of proinflammatory and inflammatory mediators

The proinflammatory mediators such as interlukin-1β (IL-1β), interlukin-6 (IL-6) and tumor necrosis factor-α (TNF- α) inflammatory mediators such as cyclooxygenase 2 (COX- 2) were estimated using the manufacturer instructions of Enzyme Linked Immunosorbent Assay kits.

### Histopathology examination

The left paw of all groups rats were cut above and below the 0.5 cm of joints. The muscle and skin of joints were trimmed away to leave the intact synovial membrane. All tissues were processed with the 3% hydrochloric acid (HCl) solution for 5–7 days, with periodic change of HCL on every 24 h for complete decalcification of joints. After that, the joints were fixed in the neutral buffered formalin (10%) for 2 days. Decalcified joints of rats were again dehydrated in different series of alcohol and joints were cleared and embedded in liquid paraffin. Decalcified joints were sliced g into 5 μm pieces with hematoxylin and eosin used for staining the tissue and preparing the slide. The slides were prepared for microscopic evaluation under light microscope (original magnification 40×, DXIT 1200, Nikon, Japan). H&E stained joint slides were examined for bone and cartilage destruction by synovial proliferation, cellular infiltration, and cartilage erosion by the following scoring system.

- **Synovial proliferation**
  For the estimation of synovial proliferation, the following score system was used. No change = Score 0; mild proliferation with 2–4 layers of synoviocytes = Score 1; moderate proliferation with four or more layers of synoviocytes, absent synovial cell invasion of adjacent connective tissue and bone with enhanced mitotic activity = Score 2; provide proliferation distinguished by adjacent cartilage and effacement of joint space, connective tissue and bone.
- **Cellular infiltration**
  Cellular infiltration: no changes: Grade 0; the small number of focal infiltrates: Score 1; extensive focal infiltration: Score 2; widespread infiltrates assaulting the capsules with combined formation: Score 3.
- **Cartilage erosion**
  No changes: Score 0; localized cartilage ruin in more than one region: Score 1; cartilage ruin: Score 2; thick cartilage ruin different locations.

### Statistical analysis

All the results were presented as mean ± SEM (standard error mean) using the one-way ANOVA {Graph Pad Prism 5.0 (Graph Pad Software, San Diego, CA, USA)}. The values of the result were considered to be significant, when the P value was *p* < 0.05, *p* < 0.01 and *p* < 0.001.

## Results

### HPTLC analysis

Various composition and amalgamations of the mobile phase were used for the required resolution of phytoconstituent (quercetin). Mobile phase solvent combination {Hexane, Ethyl acetate and formic acid (5:4:1, v/v/v)} gave a compact and dense spot. The presence of quercetin in the *MM* was confirmed by comparison of Rf value of standard quercetin. The sample bands at Rf 0.62 corresponded to quercetin (Figs. 1 and 2).

**Fig. 1:** High performance thin layer liquid chromatography (HPTLC) profiles of *Melastoma malabathricum* Linn. methanolic extract

**Fig. 2:** High performance thin layer liquid chromatography (HPTLC) profiles of Quercetin

### Molecular docking study

We have performed the molecular modeling docking studies via automated docking method into the ATP-binding site of COX-2 with s58 at 3.0 A° resolution complex (PDB code: 1cx2). The binding pose found by Maestro 9.4 for quercetin against COX-2, presented in Fig. 3. It can be observed from e molecular docking studies, that these molecules are located in such a way that the quercetin hydroxyl group creates hydrogen bond with the backbone of OH residue (Ser 530) and NH of His 90 in the hinge section. For further refinement of results, we superimposed the quercetin with s58 analyses and found the orientation of quercetin same as s58 in the COX-2 catalytic domain.

**Fig. 3:** Binding interaction of quercetin with cox2 catalytic domain (pdbid-1cx2)

For better understanding, the binding mode of quercetin at the molecular level, the molecular docking simulations of quercetin at the COX-2 catalytic ligand-binding site was carried. The Schrodinger software suite was used for the estimation of simulation. The ligand was prepared in the 3D format using the ligprep. The protein was obtained from the protein data bank (PDB ID: 1cx2), and made ready by removing the solvent, adding hydrogen and further minimization the bound ligand (s58) (Fig. 4). The re-docking study was carried for validation of co-crystal ligand parameters (s58) at the protein catalytic site, and re-docked pose was found to be 0.249 A (Fig. 5).

**Fig. 4:** Ligplot of quercetin with cox2 enzyme

**Fig. 5:** Superimposition of quercetin with s58 with cox2 catalytic domain

### Oral toxicity study

Oral administration of *MM* (500 to 2500 mg/kg b.w.) did not produce any change in the clinical or behavioral signs and symptoms, mortality or any other types of adverse reactions at the end of study. The experimental animals did not show any change in food consumption and body weight during the study period. Similar results were obtain during e subacute toxicity study, *when* compared to normal rats, confirm the safety of *MM* even upon continuous oral administration for 28 days, irrespective of the sex of rats. The results of subacute study on relative body weight of kidney (0.78 ± 0.02 g), liver (3.73 ± 0.42 g) and heart (1.98 ± 0.07 g) in male Wistar rats; and the relative body weight of kidney (0.54 ± 0.02 g), liver (2.45 ± 0.31 g) and heart (1.34 ± 0.17 g) in female Wistar rats. The relative organ weight of all *MM* (2500, 1250 and 625 mg/kg, b.w.) treated groups was almost similar to normal rats. These results indicate the body weight of normal male rats was enhanced from 140.3 ± 3.43 to 189.5 ± 8.34 with gain growth rate of 1.76 ± 0.23 and the body weight of female Wistar rats has been improved from 123.4 ± 2.83 to 156.2 ± 6.43 with 1.17 ± 0.19 growth gain rate. The body weight of *MM* (2500 mg/kg b.w.) was enhanced from 142.5 ± 6.43 to 201.2 ± 11.34 with growth gain rate 2.09 ± 0.53 and female rats treated with *MM* (2500 mg/kg b.w.) increased body weight 125.3 ± 4.32 to 161.3 ± 8.49 with 1.29 ± 0.31 growth gain rate and *MM* (1250 mg/kg b.w.) enhanced body weight from 145.8 ± 4.93 to 198.3 ± 9.76 with growth gain rate 2.1 ± 0.16 in male Wistar rats and in female Wistar rats improved the body weight 126.4 ± 3.21 to 151.2 ± 8.32 with growth gain rate 0.88 ± 0.04 per day, respectively. *MM* (625 mg/kg b.w.) enhanced the body weight 147.4 ± 2.45 to 176.3 ± 6.34 in male Wistar rats with 1.03 ± 0.03 growth gain rate and 124.6 ± 1.98 to 145.3 ± 8.23 in female Wistar rats with 0.73 ± 0.08 growth gain rate per day, respectively (Table 1).

**Table 1:** Effect of administration of *Melastoma malabathricum Linn. (MM)* (28 days) on biochemical and hematological parameters in Wistar rats (Male and Female)

S. No	Parameters	Normal control		*MM* (500 mg/kg, b.w.)		*MM* (1000 mg/kg, b.w.)		*MM* (2000 mg/kg, b.w.)	
		Male	Female	Male	Female	Male	Female	Male	Female
General effect									
1	Body Weight (gm)	189.5 ± 8.34	156.2 ± 6.43	176.3 ± 6.34	145.3 ± 8.23	198.3 ± 9.76	151.2 ± 8.32	201.2 ± 11.34	161.3 ± 8.49
2	Water Intake (mL)	102	63	83	65	94	71	104	84
3	Food Intake (gm)	52	44	32	22	44	32	54	46
Hematology									
1	RBC (10^6^/cu mm)	6.43 ± 1.21	5.11 ± 1.02	5.98 ± 1.04	5.08 ± 0.95	6.87 ± 1.65	5.21 ± 1.43	7.65 ± 1.76	5.98 ± 1.09
2	WBC (10^3^/cu mm^3^)	8.99 ± 1.43	7.21 ± 1.84	11.2 ± 1.65	9.43 ± 1.54	10.33 ± 1.64	8.65 ± 1.65	9.01 ± 1.59	7.43 ± 1.94
3	Hb (g dL^−1^)	13.01 ± 2.03	12.02 ± 2.21	12.54 ± 11.45	11.73 ± 1.98	13.06 ± 2.53	12.32 ± 2.04	14.03 ± 2.83	12.98 ± 2.47
4	Platelet (10^5^/cu mm)	4.01 ± 0.73	3.83 ± 0.49	6 ± 2.01	5.87 ± 1.84	5.21 ± 1.03	5.01 ± 1.13	4.06 ± 0.94	3.78 ± 0.73
5	Eosinophils (mm^3^)	796 ± 293	498 ± 165	598 ± 384	398 ± 194	654 ± 403	432 ± 214	731 ± 421	489 ± 283
6	Lymphocyte (mm^3^)	3990 ± 850	2983 ± 594	4350 ± 1039	3214 ± 843	4256 ± 989	3103 ± 784	4013 ± 985	3023 ± 775
7	Neutrophils (mm^3^)	1596 ± 748	1374 ± 398	1698 ± 983	1485 ± 748	1602 ± 894	1398 ± 738	1545 ± 938	1367 ± 738
Biochemical									
1	ALP (UL^−1^)	221 ± 21.83	209 ± 19.3	298 ± 31.78	285.2 ± 27.31	276.23 ± 24.54	244.5 ± 21.6	234 ± 24.5	213 ± 21.3
2	ALT (UL^−1^)	61.3 ± 2.34	50.32 ± 2.56	±	±	±	±	±	±
3	AST (UL^−1^)	103.2 ± 7.65	80.1 ± 7.87	90.3 ± 6.65	71.3 ± 8.76	95.6 ± 8.65	76.4 ± 7.54	102.3 ± 5.65	79.5 ± 6.87
4	Bilirubin (mg dL^−1^)	0.52 ± 0.09	0.36 ± 0.07	0.68 ± 0.08	0.43 ± 0.06	0.62 ± 0.06	0.41 ± 0.07	0.55 ± 0.08	0.40 ± 0.05
5	Creatinine (mg dL^−1^)	0.71 ± 0.43	0.52 ± 0.11	0.86 ± 0.22	0.64 ± 0.15	0.79 ± 0.14	0.58 ± 0.17	0.72 ± 0.21	0.54 ± 0.14
6	Urea (mg dL^−1^)	36 ± 3.21	26 ± 2.65	41.3 ± 4.54	35.1 ± 3.43	39.3 ± 3.54	32.1 ± 2.45	36.2 ± 4.32	28.5 ± 3.34
7	Cholesterol (mg dL^−1^)	71.3 ± 1.76	72.5 ± 1.54	82.6 ± 2.33	85.6 ± 3.46	79.6 ± 2.45	83.5 ± 3.43	75.3 ± 4.32	78.4 ± 3.45
8	Triglyceride (mg dL^−1^)	74.5 ± 1.87	86.7 ± 1.65	88.3 ± 1.76	89.6 ± 1.45	92.2 ± 2.43	93.3 ± 3.21	90.32 ± 2.32	92.3 ± 3.24
9	HDL (mg dL^−1^)	26.4 ± 1.41	20.6 ± 1.23	28.7 ± 2.73	22.4 ± 1.54	26.1 ± 1.83	21.3 ± 2.65	25.3 ± 2.43	20.3 ± 1.93
10	LDL (mg dL^−1^)	37.1 ± 1.23	49.83 ± 1.65	51.79 ± 2.13	60.73 ± 1.94	53.69 ± 1.86	61.91 ± 2.01	49.81 ± 1.28	58.01 ± 1.98
11	VLDL (mg dL^−1^)	14.9 ± 1.34	17.34 ± 1.67	17.66 ± 1.98	17.92 ± 1.56	18.44 ± 1.45	18.66 ± 1.76	18.06 ± 1.34	18.46 ± 1.54

The acute toxicity study did not show any significant transformation in hematological and biochemical parameters of *MM* treated rats. *MM* treated rats confirmed the proper range of hepatic and renal parameters as compared to normal rats. There was no significant alteration in lipid profile such as triglycerides, cholesterol, LDL, HDL and VLDL as compared to normal control by *MM* (Table 1).

The histology of normal and *MM* treated rats did not show any change in the appearance of the rat organs (Fig. 6).

**Fig. 6:** Histopathological examination of different vital organ of normal control and *Melastoma malabathricum* Linn. (*MM*) treated rats in sub acute toxicity study. Heart (NC): blue arrow shows the normal intercalated disc. Heart (*MM*): Black arrow depicts the normal intercalated disc. Kidney (NC): Yellow arrow demonstrates the normal tubules and glomerulus. Kidney (*MM*): Green arrow indicates the normal tubules and glomerulus. Liver (NC): Brown arrow showed the normal structure of portal and central vein of the normal hepatocytes. Liver (*MM*): Green arrow confirms the average size of portal and central vein of normal hepatocytes

### Effect of *MM* on adjuvant-induced arthritis

The rats developed the swelling and redness over 24 h after the adjuvant treatment and reached extreme intensity on day 4 (first stage of swelling developed). Consequently, redness and swelling slowly augmented until the 8^th^ day and subsequently, rats re-developed the redness and swelling. Arthritis developed during the secondary swelling, with more predominant swelling and redness, as a comparison to first stage. The secondary stage swelling was maximum by 25^th^ day of study. Pre-treatment of *MM* significantly (*P* < 0.001) censored the swelling and repressed the paw edema/redness in dose dependent manner (Fig. 7a). *MM* (500 mg/kg) showed the better recovery of the rats as compared to indomethacin treated group. Clinical assessment of rat ankles signified that the AC rats confirmed the maximum arthritis score which was considerably higher than the normal rats. AC rats treated with *MM* significantly (*P* < 0.001) produced a dose dependently inhibition of arthritic score as compared to AC rats (Fig. 7b). Considering the arthritic score, *MM* (500 mg/kg) and indomethacin significantly (*P* < 0.001) showed the better protection of rats during the arthritis, but the treatment by *MM* (500 mg/kg) was superior in comparison to indomethacin.

**Fig. 7:** Effect of *Melastoma malabathricum* Linn. (*MM*) on CFA induced arthritic rats. Arthritic was assessed in terms of enhanced of (**a**) Paw edema and (**b**) Arthritic index as described in Materials and methods. ns = non-significant, CFA = Complete Freund Adjuvant, NC = Normal Control, AC = Arthritic Control. The comparisons were made by ANOVA followed by Dunnett’s test. *P < 0.05 is considered as significant, **P < 0.01 is considered as very significant, ***P < 0.001 is considered as extremely significant

The cartilage erosion, synovial proliferation, and cell infiltration assessment between the different groups resulted in AC rats confirmed the higher score as compared to normal rats. Pre-treatment with *MM*, considerably restrained the histologic score as compared to AC group rats. Prominently, *MM* (500 mg/kg b.w.) inhibited the histologic score compared to Indomethacin group. Both *MM* (500 mg/kg) and indomethacin showed the protection/superiority over the arthritis disease but *MM* (500 mg/kg) demonstrated more superiority as compared to indomethacin group, which was confirmed by the histological observation. *MM* illustrated the average score 0.67 and indomethacin showed the average score 0.84 (Table 2).

**Table 2:** Effect of administration of *Melastoma malabathricum* Linn. *(MM)* on the scores of histopathological changes in CFA induced arthritic group rats

S. No	Histological changes	Groups				
		AC	AC + *MM* (100 mg/kg)	AC + *MM* (250 mg/kg)	AC + *MM* (500 mg/kg)	AC + Indo (10 mg/kg)
1	Synovial proliferation					
	Grade 0	-	-	-	2	1
	Grade 1	-	-	-	-	1
	Grade 2	-	2	2	2	2
	Grade 3	5	2	1	-	-
	Total	15	10	7	4	5
	mean	3	2.5	2.3	1	1.25
2	Cartilage erosion					
	Grade 0	-	-	2	4	3
	Grade 1	-	2	2	1	1
	Grade 2	2	1	-	-	-
	Grade 3	3	-	-	-	-
	Total	13	4	2	1	1
	mean	2.6	1.33	0.50	0.20	0.25
3	Cellular infiltration					
	Grade 0	-	-	-	3	3
	Grade 1	-	1	2	2	1
	Grade 2	-	2	2	1	2
	Grade 3	5	1	-	-	-
	Total	15	10	6	4	5
	mean	3	2.5	1.5	0.67	0.84

Body weight declined in AC rats at the end of experimental study (Fig. 8). AC rats treated with *MM* and Indo significantly (*P* < 0.001) improved the body weight in dose dependent manner. (Fig. 8).

**Fig. 8:** Effect of *Melastoma malabathricum* Linn. (*MM*) on CFA induced arthritic rats. Arthritic was assessed in terms of alteration of body weight as described in Materials and methods. ns = non-significant, CFA = Complete Freund Adjuvant, NC = Normal Control, AC = Arthritic Control. The comparisons were made by ANOVA followed by Dunnett’s test. *P < 0.05 is considered as significant, **P < 0.01 is considered as very significant, ***P < 0.001 is considered as extremely significant

### Effect of *MM* on hematological parameters

CFA made a compelling upsurge in fructification of WBC (8 ± 0.32 cells/cu.mm). The *MM* treatment conferred important protection from the same, just about consistently (Fig. 6). Similarly, outstanding enhancement of ESR was noted in AC control (14 ± 0.46 million/cu.mm (gm%) in counterpart to normal control (9.8 ± 0.29 million/cu.mm (gm%). Concomitant administration of *MM* significantly (*P* < 0.001) altered the WBC and ESR. Compelling subsidence in the hematological parameters of RBC as perceived in AC (4.4 ± 0.25 million/cu.mm). Similarly, the outstanding decline in Hb was noted in AC (9.6 ± 1.37 cells/cu.mm) in counterpart to normal control AC (13.6 ± 0.54 cells/cu.mm), it is notable that treatment with *MM* helped to restore the hematological parameters of RBC and WBC synchronously (Fig. 9).

**Fig. 9:** Effect of *Melastoma malabathricum* Linn. (*MM*) on CFA induced arthritic rats. Arthritic was assessed in terms of modulation of (**a**) WBC, (**b**) RBC, (**c**) Hb and (**d**) ESR as described in Materials and methods. ns = non-significant, CFA = Complete Freund Adjuvant, NC = Normal Control, AC = Arthritic Control, WBC = White blood cell, RBC = Red blood cell, Hb = Hemoglobin, ESR = Erythrocyte sedimentation rate. The comparisons were made by ANOVA followed by Dunnett’s test. *P < 0.05 is considered as significant, **P < 0.01 is considered as very significant, ***P < 0.001 is considered as extremely significant

### Effect of *MM* on antioxidant enzymes

We also examined the antioxidant parameters (Fig. 10). As expected, CFA treatment considerably increased the MDA enzyme activity and decreased the activities of SOD, GSH and GPx. AC rats treated with *MM* significantly (*P* < 0.001) altered the antioxidant enzymes to near the normal rats in dose dependent manner.

**Fig. 10:** Effect of *Melastoma malabathricum* Linn. (*MM*) on CFA induced arthritic rats. Arthritic was assessed in terms of modulation of (**a**) MDA, (**b**) GPx, (**c**) SOD and (**d**) GSH as described in Materials and methods. ns = non-significant, CFA = Complete Freund Adjuvant, NC = Normal Control, AC = Arthritic Control, MDA = Malonaldehyde, GPx = Glutathione peroxidase, SOD = Superoxide dismutase, GSH = Glutathione. The comparisons were made by ANOVA followed by Dunnett’s test. *P < 0.05 is considered as significant, **P < 0.01 is considered as very significant, ***P < 0.001 is considered as extremely significant

### Effect of *MM* on inflammatory mediators

The levels of COX-2, IL-6, TNF-α and IL-1β were augmented in the serum after CFA treatment. AC rats received oral administration of *MM* apparent supplementary increase of the same (Fig. 11).

**Fig. 11:** Effect of *Melastoma malabathricum* Linn. (*MM*) on CFA induced arthritic rats. Arthritic was assessed in terms of modulation of proinflammatory mediators such as (**a**) TNF-α, (**b**) IL-6, (**c**) IL-1β and (**d**) COX-2 as described in Materials and methods. ns = non-significant, CFA = Complete Freund Adjuvant, NC = Normal Control, AC = Arthritic Control, TNF-α = Tumor necrosis factor-α, IL-6 = Interlukin-6, IL-1β = Interlukin 1β. The comparisons were made by ANOVA followed by Dunnett’s test. *P < 0.05 is considered as significant, **P < 0.01 is considered as very significant, ***P < 0.001 is considered as extremely significant

### Effect of *MM* on histopathology of CFA-induced rats

The histopathology observation of normal control and CFA-induced rats are showed in Fig. 12. The normal rat histopathology explained clean articular surface among 1–4 layers of synovial cells and normal articular smooth surface with a loose connective tissue. This also contained the fatty tissue below the synovial membrane. AC control rat histopathology showed the hyperplasia in the articular region with the loose connectivity of tissue. The synovial defect showed the distortion of pannus formation of bone and cartilage. The deformity of the joint was widespread resulted due to increased sizes and connectivity of synovial membrane. AC showed the loose arrangement of connectivity of tissue due to hyperemia, edema and infiltration with provocative cells (Fig. 12b). AC rats treated with *MM* showed the remarkable restoration of all histology characteristics in dose dependent manner. *MM* dose (500 mg/kg b.w.) displayed enhanced histopathology as compared to *MM* dose (100 and 250 mg/kg b.w.) (Fig. 12 c-e).

**Fig. 12:** Histopathological effect of *Melastoma malabathricum* Linn. (*MM*) on CFA induced arthritic rats. **a** Normal Control: showed the normal architecture of articular cartilage; **b** AC control: showed the bone erosion, mononuclear cell infiltration and deformity of the bone with the presence of leukocytes infiltration (*red arrow*) and synovitis (*blue arrow*); **c** AC control + *MM* (100 mg/kg b.w.) showed the leukocytes infiltration (*black arrow*) and synovitis (*yellow arrow*); **d** AC control + *MM* (250 mg/kg b.w.) showed the leukocytes infiltration (*black arrow*); **e** AC control + *MM* (500 mg/kg b.w.) confirmed the normal architecture with less deformity of bone and cartilage; **f** AC control + Indo (10 mg/kg b.w.): treatment rats demonstrated the recovered histopathological profile towards normal architecture with less deformity of bone and cartilage

## Discussion

Arthritis is a chronic painful inflammatory disease, affecting more than 1% population in developed countries. On the basis of biochemical markers, CFA-induced arthritis is clinically classified into four phases, initial phase developed during the first week after injecting the CFA with acute local inflammation and having some effects on liver; in the second week afterward, extend the reduction of acute inflammation and start the periarteritis; third-fourth week develops the arthritis with chronic inflammation, osteogenic and periarteritis activity, therefore, the fifth week onwards (forever), with permanent articular deformity and minimal inflammation [33, 34].

Our study showed the credible protecting impact of this plant against the chronic inflammation induced by CFA. The results confirmed the use of *MM* extract as an antiarthritic agent in Indian folk medicine on the scientific basis. The conclusion of this study clearly explains that the *MM* extract is a potent antiarthritic remedy against chronic phases of inflammation. Topical and systemic application of *MM* is commonly observed for the treatment of inflammation, predominantly, arthritis (ama vata) which has been pursued for many years in the practice of Indian system of medicine (Ayurveda).

*MM* extract is a rich source of the flavonoids (quercetin). Flavonoids play an important role to inhibit the inflammation via apoptotic mechanism (calcium dependent) or cyclin-dependent kinase inhibitors; modify the cell cycle capture at the G1/S phase (Extracellular growth signals stimulate progression through the first gap phase G1, and into S, where genomic DNA is replicated); inhibit the cell-survival kinase and the inflammatory transcription factors; down-regulate the antiapoptotic gene products [34, 35].

The CFA-induced arthritis model is the most extensively use model to investigate the clinical and pathogenic changes, which are similar to human arthritis [25]. Further this method helps in determining the correlation between efficacy of therapeutic agents and RA model [36, 37]. The adjuvant-induced inflammatory process involves fenestration of microvasculature, leakage of element into the interstitial space and passage of macrophages, lymphocytes into inflamed tissue; where adjuvant inoculation releases the number of inflammatory mediators like cytokines, histamine, 5 hydroxytryptamine, bradykinin, various chemotactic factor, interferons and prostaglandin into inflamed area. These mediators are liable for demolition and destruction of bone, cartilage and associated with pain, which can lead to several disabilities. Other mechanisms involves leukocytes and phagocytes, preparing a complex with the mediators, releasing the lysosomal enzymes and causing the injury of cartilage and other tissue. CFA affected the soft tissue and created the swelling near the ankle joints confirm the expansion of arthritis which was measured as edema of the particular tissues [38, 39]. In the current study, the efficacy of *MM* treated rats was evaluated in the proliferative phase of inflammation, showing the minimization of the chronic swelling induced by CFA. The first indication of the antiarthritic effect of *MM* was observed when the administered extract (100, 250 and 500 mg/kg) showed a significant dose-dependent reduction of paw edema with 59.17%, 74.16%, and 87.72%, as compared to AC rats respectively. However, *MM* received rats did not show enhancement of joint diameter, which suggests that mechanisms involved, is inhibition of inflammatory autacoids. The most likely mechanism for *MM* extract may be inhibition of proinflammatory mediators, which could have lead to an alteration in the immunological situation during the delayed phase of the response. The determination of body weight and foot thickness of CFA-induced arthritis animals has been used to evaluate the antiarthritic effect of drug treatment. We found increased body weight of rats with decreased thickness of rat paw as compared to AC rats.

AC rats confirmed the decline level of RBC, Hb and increased levels of WBC, ESR. WBC is an important component of an immune system which is associated with induction of inflammation and is related to other infectious diseases [40]. During the arthritic condition, 1 L-1β mediated increase in WBCs, cause the growth of colony stimulating factors and production of inflammatory macrophages and granulocyte [41]. *MM* treated rats significantly suppressed the migration of inflammatory macrophages and granulocytes in dose dependent manner. On the other hand, increased ESR levels start the generation of endogenous proteins (fibrinogen, α/β globulin) and indicate the disease progression [42]. During the arthritic condition, decreased levels of RBC and Hb, associated with anemic condition due to erythrocyte deformability (shorten the life span of erythrocytes), which result in declined level of RBC during arthritis [43, 44]. It is projected that the declined levels of Hb during arthritis, results in reduction of erythropoietin level (decreased the level of bone marrow erythropoietin level) and premature destruction of RBCs [28, 45]. Restoration of hematological parameters to normal by MM extracts supports its anti-arthritic effect.

ROS/RNS/free radical incessantly formed inside the body as a consequence of exposure to many endogenous and exogenous chemicals. There is equilibrium between the antioxidants and generated ROS/RNS, as the generation of ROS/RNS is stabled by endogenous antioxidants. Any disparity among the inactivation and production of ROS/RNS species leads to cellular dysfunction and unwanted pathological conditions including RA [46]. The ROS/RNS species start the deprivation of synovial fluid and induce the depolymerization of hyaluronic acid which turns the loss of viscosity in joints [47]. The human body has an efficient mechanism to avoid and deactivate the free radical generation/production damage caused by endogenous antioxidants such as SOD, GSH, GPx and CAT. SOD is metalloprotein that is the first line antioxidant marker involve in antioxidant defense. Decreased levels of RBCs in arthritic conditions increase the production of superoxide (O_2_) and hydrogen peroxide radicals (H_2_O_2_) due to accumulation of inflammatory macrophages and granulocytes in the inflamed area [47, 48]. Lipid peroxidation (LPO) is a common feature of rheumatic arthritis. MDA (as an indicator of lipid peroxidation) is used to evaluate the LPO. MDA is a pro-oxidant factor which determines the oxidative stress present in the rats [48]. AC rats showed increased levels of MDA as compared to NC rats, due to elevated d level, it also started the accumulation of neutrophils in the inflamed area. CFA-induced arthritic rats that received *MM* significantly (*P* < 0.001) declined the levels of MDA. GSH and SOD are the first line antioxidants against scavenging the free radicals. SOD coverts the superoxide radical to H_2_O_2_ and is widely used to protect the cell damage during the toxic effects of O_2_ anion. First line antioxidants catalytically scavenge the hydrogen peroxide (H_2_O_2_) and superoxide (O_2_-) molecules. Endogenous antioxidant GPx reduced the H_2_O_2_ in the presence of GSH to form oxidized glutathione and water [49]. CFA-induced arthritic rats that received *MM* had significantly (*P* < 0.001) modulated the level of an antioxidant enzyme as compared to AC rats.

Many researchers have shown that the proinflammatory mediators play a crucial role in the pathogenesis of arthritis [50]. TNF-α (pleiotropic inflammatory cytokines) plays a crucial role in pathogenesis of acute and chronic inflammation, associated with the neutrophils and lymphocytes in endothelial cells via inflamed tissue. TNF-α, present in sera and synovial fluid of arthritic patients is a laboratory and clinical marker for estimation/confirmation of RA disease [51–53]. It also promotes the generation of macrophage chemotactic protein-1 (MCP-1), IL-6 and IL-1β, which are involved in increasing the inflammatory reaction. Macrophages release the proinflammatory IL-1β, which enhances the inflammatory reaction. Both inflammatory cytokines (IL-1β and TNF-α) activated through the osteoclasts and nuclear factor are responsible for re-absorption and obliteration of bones. The generation of proinflammatory cytokines such as IL-6 starts through the T-cells, fibroblasts and monocytes, which initiate the induction of osteoclast discrimination and stimulates the MCP-1. All these proinflammatory cytokines are also involved in enhancing the clinical sign of arthritis and expansion of arthritic symptoms as well as body weight loss and joint swelling [25, 27]. In the current study, we observed a considerable enhancement of serum TNF-α, IL-1β and IL-6 concentrations in AC group as compared to NC group. Treatment with *MM* decreased the serum levels of IL-1β, TNF-α and IL-6 without disturbing other inflammatory mediators.

## Conclusion

In conclusion, *Melastoma malabathricum Linn* was effective in attenuating the CFA-induced arthritis rats in a dose-dependently manner, and therefore it could be investigated as a probable treatment for chronic arthritis conditions in humans. The results obtained from the current study confirm the use of *MM* extract in traditional Indian medicine for the management of painful inflammatory and arthritic conditions. Additional work is going on to isolate, characterize and identified the structure of phytoconstituents responsible for the antiarthritic activity.

## Highlights

*Melastoma malabathricum* Linn reduced CFA induced activation of the proinflammatory cytokines.

*Melastoma malabathricum* Linn reduced the CFA induced activation of COX-2.

*Melastoma malabathricum* Linn significantly suppressed the paw edema.

*Melastoma malabathricum* Linn modulation the CFA induced antioxidant parameters.

## Abbreviations

AC: Arthritic control
ALP: Alkaline phosphatase
ALT: Alanine transaminase
AST: Aspartate aminotransferase
b.w.: Body weight
CAT: Catalase
CFA: Complete Freund’s adjuvant
CMC: Carboxyl methyl cellulose
COX-2: Cyclooxygenase 2
DNA: Deoxyribonucleic acid
ELISA: Enzyme Linked Immunosorbent Assay
ESR: Erthrocytes sedimentation rate
GPx: Glutathione peroxidase
H: Hour
Hb: Hemoglobin
HCl: Hydrochloric acid
HDL: High-density lipoprotein
HPTLC: High-performance thin layer chromatography
IL-1β: Interlukin-1β
IL-6: Interlukin-6
Indo: Indomethacin
Kg: Kilogram
LDL: Low-density lipoprotein
LPO: Lipid peroxidation
MCP-1: Macrophage chemotactic protein-1
Mg: Milligram
MM: *Melastoma malabathricum Linn*.
NSAIDs: Nonsteroidal anti-inflammatory drugs
O_2_: Superoxide
RA: Rheumatoid arthritis
RBC: Red blood cells
RNS: Reactive nitrogen species
ROS: Reactive oxygen species
SEM: Standard error mean
SOD: Superoxide dismutase
TLC: Thin layer chromatography
TNF- α: Tumor necrosis factor-α
VLDL: Very low-density lipoprotein
WBC: White blood cells
